The article "The Subject Construction and Role Mental Model Construction of Erotic Movies Based on Lacan's Desire Theory" was retracted in 2024. Reasons: signs of a paper mill; suspected computer-generated content; unreliable results or conclusions; concerns about the data.

# The Subject Construction and Role Mental Model Construction of Erotic Movies Based on Lacan's Desire Theory

**DOI:** 10.1155/2022/7751995

**Published:** 2022-06-13

**Authors:** Shuqin Feng

**Affiliations:** Southwest Jiaotong University, Chengdu, Sichuan 611756, China

## Abstract

Jacques Lacan is a famous French psychoanalyst, but his influence has long gone beyond the scope of psychoanalysis and has affected almost all fields of “human science.” Film and psychoanalysis coincided almost simultaneously and influenced each other. But with the development of film, researchers found that film studies in the period of classic film and film semiotics have come to an end. It has certain theoretical value to explore the construction of the subject and the mental model of the erotic film based on Lacan's desire theory. *Method.* The body in the film and video described in this paper includes both the material body as an aesthetic object and the spiritual body with aesthetic consciousness. The so-called artistic presentation of the body element means that the beauty of the body form displayed by the actor's body in the film video is perceived by the audience, and the desire to stare is captured by the audience, thereby completing the audience's entire body composed of eyes, body, and mind. The body is not only an aesthetic object but also an aesthetic subject, and the human cognitive system is not just a closed brain. Because the nervous system, body, and environment are constantly changing and interacting, true cognition is a unified system of all three. The main part of this paper uses Lacan's psychoanalytic theory to deeply analyze the relationship between the characters shown in the film. From the cognitive impairment of the self to the failure of communication between characters, the language of uncertainty entangled by desire is removed, and the behavior and facial expressions of the movie characters are used as the analysis basis to fully interpret the inner world of the characters. This includes love, hatred, pain, struggle, and many other contradictory emotions. In addition, this paper also analyzes the metaphor of the relationship between the characters from the perspective of semiotics and discusses the description of the relationship between the characters from the lens language from the perspective of cinematography. The special meaning conveyed by the recurring elements in the film is emphasized, and the correlation between the pictures is explained from the less mentioned photographic aspect of the film. *Results/Discussion.* Looking at Lacan's theory, the subject, the other, and desire are linked by the subject spirit, which is the core of the connection between the three, and only through the resistance and struggle of the subject spirit can the illusion of the subject be broken. Bewilderment and the suppression of the other and desire finally become the self. And the embodiment of this true self is particularly prominent in film art. Lacan's purpose is not merely to dissolve the subject but to seek a stand in the midst of destruction, pursuing the ultimate transcendence of man's desire for the external other and internal desire.

The article "The Subject Construction and Role Mental Model Construction of Erotic Movies Based on Lacan's Desire Theory" was retracted in 2024. Reasons: signs of a paper mill; suspected computer-generated content; unreliable results or conclusions; concerns about the data.

## 1. Introduction

With the emergence of Lacan's theory, people began to think about all kinds of “people” in a new way. Although Lacan's theory is complex, it is generally constructed with his mirror image theory as the cornerstone and language as a tool [1]. As a construct of human culture, film is a kind of visual culture, which is deeply influenced by Lacan's mirror image. The book “Contemporary Film Analysis” is devoted to the special state of film analysis of psychoanalytic theory, and they argued that the Freud-Lacanian psychoanalysis is more concerned with the production of meaning and also pointed out that before the emergence of the second semiotics of Metz's film, film theory was very cautious in the use of psychoanalysis [2]. But by the early 1990s, many structuralist film semioticians were enthusiastic about formalist structural analysis, and they began to move psychoanalysis from the astray of scientific rationalization to a new one based on culture and anthropology.

In a certain sense, man is the embodiment of desire, and the difference between man and animal is also reflected in the difference in desire between the two [3]. The desires of animals are generally manifested in instinctive desires: the desire for survival, the desire for food and clothing, and so on; while human beings are different, their desires must be absolutely higher than the desires of animals [4]. To be man, in order for man to be essentially and practically different from animals, man's desires must in fact transcend his animal desires. However, desire is ultimately a desire for a value. For an animal, the highest value is its own life. All the desires of animals are closely linked with the desire to preserve life [5]. And human desires go beyond this desire to preserve life. In other words, a man truly becomes a man only when his desires are separated from his desire only for survival.

The essence of “recognition” is the desire of the subject to desire the other, and what the subject wants is exactly what the other person wants, and what both the subject and the other want is to be “recognized” [6]. The desire to desire another is to hope that the value of what I am or what I “represent” is the value that the other desires [7]. The achievement of mutual recognition is impossible in a master-slave relationship. Lacan's proposition that “the desire of man is the desire of the other” is obviously influenced by this kind of “recognition” between subjects [8, 9].

The article "The Subject Construction and Role Mental Model Construction of Erotic Movies Based on Lacan's Desire Theory" was retracted in 2024. Reasons: signs of a paper mill; suspected computer-generated content; unreliable results or conclusions; concerns about the data.

We extend the scope of the nervous system theory of the aesthetic subject to the whole body, because the whole body exists and is generated as an aesthetic cognitive module [10]. That is to say, we do not “own” a body, but our body constructs an aesthetic cognition module with the systematic thinking of “existence,” in order to achieve the aesthetic cognition of the body presented in the film and video. The effect is as follows: at first glance, it is a body that is “flesh,” then when you look at it again, it is a body that is “I want” and is in the world, and when you look at it again, it is an aesthetic body that is conscious of “I can” [11, 12].

The interpretation of the film in this paper does not just stop at revealing the theme of the film, but based on the principle of similar style and consistent theme, using psychoanalytic theory to show the theme of the director and actors, and to deepen the relationship between the characters portrayed in the film. The secrets of human nature and the soul discussed in the film are certainly worth thinking about, but the way the film presents the theme also requires attention. How can these metaphysical problems recur in literary works and endure human beings and how can they be unique in Bergman's work? It is so vivid and thought-provoking under the film lens.

Through the analysis of Lacan's theory, we understand that the subject is not only facing the danger of being swallowed up by his own illusions but also being suppressed by the other and his desires, making the subject itself like Freud's “self.” However, the subject itself has a potential ability enough to make the subject achieve itself, that is, the subject spirit. Although Lacan did not explicitly put forward this concept, we can realize from his words that he respects and maintains the value of the subject. The people who warned us and told us how to save the spirit of the subject were about to be wiped out by this materialistic and down-to-earth “waste” society.

## 2. Methods

### 2.1. Analysis of the Beauty of the Construction of Film and Video Subject

#### 2.1.1. The Aesthetic Connotation of Subject Construction

The body is not only an aesthetic object but also an aesthetic subject. The human cognitive system is not just a closed brain. Since the nervous system, the body, and the environment are constantly changing and interacting, the real cognitive system contains three unified system. Therefore, the body and the brain must work together to complete aesthetic activities. Somaesthetics has two basic characteristics, “one is that it pays attention to the mind and body of the people in the world, and the other is that it pays attention to the desire for the beauty and power of the body itself.” The fundamental characteristic of the body that distinguishes it from the mind is that it must occupy a specific space and must have an uninterrupted and healthy exchange of energy with the environment. This article basically fully reflects the three levels of the somaesthetics picture. The subject in the movie image (the actor's flesh) is the aesthetic object, the audience's body is the aesthetic subject, and the process of watching a movie is an embodied aesthetic activity. By incarnation, we mean the biological and physical presence and presence of our bodies, which are preconditions for subjective emotion, language, thought, and social interaction.

The article "The Subject Construction and Role Mental Model Construction of Erotic Movies Based on Lacan's Desire Theory" was retracted in 2024. Reasons: signs of a paper mill; suspected computer-generated content; unreliable results or conclusions; concerns about the data.

The study of incarnation and the beauty of film and video is to affirm the role of human existence and superstructures such as morality and culture in condensing our beautiful soul. The connection between nature and human beings, matter and meaning is morality. It can be said that the moral body is where the value of our materiality and meaning meet. It is through the moral nature of the body (including pleasure) that we can connect with cultural politics. The body is presented in the form of artistic images, and the purpose of presentation is to express and display [13]. At first, we thought that the expressiveness of the body is entirely due to the perceptual patterns formed by the form and structural composition of the body. After the intervention of cognitive neuroscience and brain science, we have a deeper understanding that these feelings come not only from aesthetic objects but also from aesthetic subjects. The function of the nervous system, that is, aesthetic activity, is a spiritual phenomenon, but it has an irrefutable physiological basis [14]. Representativeness is not really conveyed by these “geometric-technical” properties of the perceptual objects themselves, but by the forces that these properties evoke in the viewer's nervous system. Only when there is a “tentative tension” or “movement” can they be perceived as expressive [15].

Film actors are the main body of performance in film and video, and they are also the most active elements in the entire film art. Actors rely on their bodies to “shape” their performances, so that the performance has a “tendency”, so as to maximize the “expressiveness” of the body [16]. Only when the limit is presented will this force affect our emotions. Regarding the understanding of expressiveness, Rudolf Einham once said in his book “Art and Visual Perception” that “expressiveness depends on the basic nature of perception that we experience when we perceive a particular image [17, 18]. Expressivity takes on a deeper meaning when we recognize that these dynamic qualities signify a certain human destiny. One of the factors that can produce the form perception mode or aesthetic activity is that the object to be aesthetic needs to be expressive; that is to say, it conveys “tendency tension” [19].

The article "The Subject Construction and Role Mental Model Construction of Erotic Movies Based on Lacan's Desire Theory" was retracted in 2024. Reasons: signs of a paper mill; suspected computer-generated content; unreliable results or conclusions; concerns about the data.

#### 2.1.2. The Role of Formal Perception Mode in Subject Construction

The body is the easiest and most direct way to show love and hate, especially in the visual image system of film. At the same time, the understanding of subject construction in film and television requires the participation of our nerve cells, and the aesthetic cognition module can help us to understand the beauty of subject construction more deeply. Now, briefly explain what cognitive modules mean in cognitive aesthetics; just like modules in design terminology, there are similar modules in our human brains. To put it another way, the reason why we can design the physical structure of a module is precisely because we already have such an organic structure in our brains, which is a process from matter to thought and then to material realization.

For an object to be aesthetic, whether it will trigger our sense of beauty or not depends on the inner working state of our aesthetic subject at that time. Modern cognitive science finds: “Human reasoning arises from a kind of animal reasoning, which is closely related to the special structure of our bodies and brains; the human body, brain, and interaction with the environment provide the unconscious basis for everyday speculation” [20]. Most fruits and foods are round or close to round, which is of course due to the wind or the earth, water, etc., so that it needs a round shape to resist external forces, and over time, we have a special sense of circle. At the same time, because the circle is not easy to hurt us, and remember the shape of this object, the input module is constantly strengthened.

### 2.2. Aesthetic Acceptance of Subject Construction in Film and Video

There is an unavoidable basic question in our research on aesthetic activities: how can the appreciation and perception of beauty be universal and inevitable without relying on a priori aesthetic judgment? So Kant put forward a concept-aesthetic sense of commonality. Kant's view of the common sense is: “We must understand the common sense as an idea of a common feeling, that is, an idea of the ability to judge, which in its own reflection takes into account the thinking of every other person in the in order to present his judgments as if they were dependent on all human reason, and thereby avoid the illusion that would adversely affect judgments from subjective private conditions that might easily be seen as objective.” This explanation effectively avoids the whirlpool of subjectivity and places feeling and judgment at an anthropological level. Although Kant's interpretation of aesthetic common sense may have unverifiable places, its philosophical thinking and human developmental thinking is very important.

The article "The Subject Construction and Role Mental Model Construction of Erotic Movies Based on Lacan's Desire Theory" was retracted in 2024. Reasons: signs of a paper mill; suspected computer-generated content; unreliable results or conclusions; concerns about the data.

The personal unconscious depends on a deeper level, which is neither derived from personal experience nor acquired, but innate. We call this deeper level the collective unconscious.

The term “collective” was chosen because this part of the unconscious is not individual but universal; unlike the individual psyche, its content and patterns of behavior are largely the same everywhere and in all individuals. In other words, it is indistinguishable from all people and thus constitutes a common psychological basis of transpersonality that pervades us all.

### 2.3. Lacan's Psychoanalysis

#### 2.3.1. Self-Knowledge in the Initial Stage of the Subject: The Mirror Stage

Lacan's mirror stage is based on Walloon's “mirror experiment” in child psychology research. Lacan believes that the mirror stage is an important turning point in an infant's life, and it is also a period in which everyone's self-identity is initially formed. Babies between six months and eighteen months need to rely on the hold of others to see their own mirror images. At this time, they cannot distinguish themselves from the image of their mother or the other. Babies confuse the self with the other. Later, with the increase of the baby's body movements, he was gradually able to recognize his own image in the mirror image and at the same time distinguish the other from himself. The baby sees the image of the mother holding him and the familiar family environment around him in the mirror, which makes the baby more sure of himself in the mirror. Lacan further pointed out that in the self-identification of the subject in the process of growth, the mirror image is not only limited to the real mirror but also includes the reflection of the subject contained in the eyes of others around him.

#### 2.3.2. The Subject Object of Psychoanalysis: Intersubjectivity

The subject is a knower and an actor, and the self-knowledge function mentioned above is one of the most important cognitive functions of the subject. The subject can always reach others through the function of self-knowledge. Intersubjectivity refers to the mutual relationship and interaction between subjects. Lacan believes that intersubjectivity determines the nature of subjects, and the main activity that maintains the relationship between subjects is the activity of referring to things and conveying meaning between subjects; that is, the use of language is the essence of intersubjectivity. In this way, Lacan introduces language into psychoanalysis.

The article "The Subject Construction and Role Mental Model Construction of Erotic Movies Based on Lacan's Desire Theory" was retracted in 2024. Reasons: signs of a paper mill; suspected computer-generated content; unreliable results or conclusions; concerns about the data.

### 2.4. Role Mental Model

#### 2.4.1. Human Cognitive Process

Information processing cognitive psychologists believe that human cognitive process is the process of information integration and information processing. The human cognitive process is regarded as a system for processing information. This system is very similar to the computer processing system, which is a process of information input-processing-output. The cognitive process of the subject of erotic movies consists of a set of closely continuous cognitive stages, including the acquisition, encoding, storage, extraction, and use of external information, as shown in Figure 1.

The function of human senses is to obtain external information. The acquisition of information is that humans themselves accept external stimulus information that directly acts on the senses; the encoding of information is that humans themselves convert one form of external information into another form of information. The storage of information means that humans store the encoded information for later extraction and use; the extraction and use of information means that humans extract the previously encoded and stored information under the action of corresponding external stimuli. In this process, new information will be acquired, encoded, and stored, so the human cognitive process has dynamic development. For individuals, different individuals have corresponding external information and coding methods in their cognitive activities.

#### 2.4.2. Construction of the Role Mental Model

Mental models are the knowledge that exists in the user's mind about the concepts and behaviors an erotic movie should have. This knowledge about the concept and behavior of erotic movies may be derived from the user's previous experience with similar erotic movies, or a user's expectation of erotic movie concepts and behaviors based on the goals to be achieved by using the erotic movie. From Donald Norman's definition of mental model, we can infer three sources of the role's mental model: experience with erotic movies, expectations of erotic movie concepts, and expectations of erotic movie behavior. Erotic movie concept expectations and erotic movie behavior expectations are summarized as users' expectations for erotic movies. Therefore, the source of the role mental model is summarized in two aspects, that is, the experience of erotic movies and the expectations of erotic movies.

The article "The Subject Construction and Role Mental Model Construction of Erotic Movies Based on Lacan's Desire Theory" was retracted in 2024. Reasons: signs of a paper mill; suspected computer-generated content; unreliable results or conclusions; concerns about the data.

The user's mental model is often based on the accumulation of the user's real-life experience. The user's mental model will change with the changes of time, living environment, values, and other factors. The role mental model has the characteristics of dynamic development and change, corresponding to the role mental model, and characteristics of assimilation and adaptation. When the user is using a new erotic movie, that is, the user receives a new stimulus from the outside world, the user's mental model will undergo a dynamic change process of assimilating or adapting to the new knowledge.

Assimilation of new knowledge means that the user uses the existing experience and knowledge to successfully complete the operation of erotic movies, completes the user's established goals, and makes the original role mental model to be strengthened and developed.

Adapting to new knowledge refers to a gradual learning process in which the target user's own original experience cannot fully guide the user to use the new interactive function of erotic movies smoothly, and users operate through their own learning and exploration, thereby obtaining feedback on erotic movies. In this process, users learn new experiences and research methods and finally complete the goals set by users. The new understanding gradually replaces the user's existing experience and understanding and then evolves into a new role mental model.

### 2.5. Analysis Method of Role Mental Model

In order to better match the performance model of the mobile collaboration software with the target user's mental model, the designer's first job is to analyze the target user's mental model. So, what method is used to analyze the role mental model? Adopting a user-centered analysis method can facilitate the analysis of role mental models.

Task analysis splits erotic movies into a series of subtasks to understand the user's goals, tasks, strategies, steps, and usage. The causal relationship analyzes a certain connection between the user's cognitive habits and hypothetical things to understand the reasons for the user's behavior.

Mental models are the knowledge that exists in the user's mind about the concepts and behaviors an erotic movie should have. This knowledge may come from the user's previous experience with similar erotic movies, or a user's expectation of erotic movie concepts and behaviors according to the goals to be achieved by using the erotic movie. The analysis of the role mental model can start from the knowledge source of the mental model. On the one hand, the user's model comes from the experience of using existing erotic movies, and on the other hand, it comes from the user's expectation of the concept and behavior of new erotic movies.

The article "The Subject Construction and Role Mental Model Construction of Erotic Movies Based on Lacan's Desire Theory" was retracted in 2024. Reasons: signs of a paper mill; suspected computer-generated content; unreliable results or conclusions; concerns about the data.

## 3. Results

### 3.1. The Influence of Lacan's Unconscious on the Subject

The unconscious language structure affects the subject, and the subject symbolically resides in the structure of the signifier and is in the position of the other with a structure of lack. The subject becomes the subject of the signifier, the subject of the other. At the same time, the subject also loses its own origin and image in the chain of signifiers, obscuring its own essence. Therefore, the subject can only find its own essence in the overlapping of signifiers. At this time, the subject is separated from its essence, and this separation is a separation of the subject and the subject. In essence, the subject is detached from the subject.

In the unconscious language structure, the subject is in the grand objective communication structure, and the subject begins to be objectified and alienated. At this time, the development of the subject goes far beyond the individual's subjective feelings, the subject begins to be constructed, and the subjectivity is gradually forgotten. The subject gradually becomes a subject detached from subjectivity. Lacan also mentioned the subject and subject in “The Role and Field of Speech and Language in Psychoanalysis.” According to his theoretical point of view, subjectivity is the postorganization of the subject through the instinctual stage. From the analysis of the development stage of the subject, the instinct stage of the subject is followed by the symbolic stage. Thus, subjectivity is organized in the symbolic phase of the subject. When the subject is in the symbolic stage, it is in the unconscious language structure, and the subjectivity is hidden by the symbolic signifier structure. He believes that subjectivity, as the internal driving force of the subject, drives the subject to record its activities and behaviors in the form of success or failure, and gives the subject's desire expression different meanings; the subject's desire can be satisfied in different forms. The influence of Lacan's unconscious on the subject is shown in Figure 2.

Lacan believes: “The subject goes far beyond what the individual ‘subjectively' feels. He can always reach the truth, and he will come out of your closed mouth.” Combining his theoretical analysis of the structure of unconscious language, Lacan puts the subject in the whole unconscious language structure; his subject exists in the whole symbol system and is the unconscious subject.

The article "The Subject Construction and Role Mental Model Construction of Erotic Movies Based on Lacan's Desire Theory" was retracted in 2024. Reasons: signs of a paper mill; suspected computer-generated content; unreliable results or conclusions; concerns about the data.

This subject is beyond the individual consciousness, the existence form of the unconscious language, and the symbol of the other. The “other” itself is an alien force outside the individual, not something that belongs to the individual's subjective feelings.

Therefore, the unconscious subject is the subject of the other, and the subject of the other is a subject detached from personal subjectivity.

To sum up, the subject under the influence of Lacan's unconscious language structure becomes the unconscious subject, becomes the subject of the other, and is a subject separated from the individual subjectivity.

### 3.2. Motives of Desire: The Effect of Residual Pleasure Objects on the Subject

The motivation of desire is that in the return of the original pleasure, “all the objects of the subject's desire are the remnants of some kind of original pleasure experience”, in the moment we smell the sweet taste and the moment we hear the beautiful sound. In a flash of beauty, all this points to the original pleasure, the child's desiring relation to the mother, the oneness with the mother, and the unity of me and the other. This unspoken yet clearly felt return to the original pleasure is what motivates our desire. However, this return to the original pleasure is not embodied in our demands in a direct way; it is embedded between reality, imagination, and symbolism, and it is not a complete return, but a surplus of pleasure. It is the surplus of pleasure because it has no use value in itself and cannot be represented by any symbol.

The remainder of this pleasure is the moment when the subject melts into the other and will always be a moment. Just as the child becomes the center of the other in the board game, this state can only be temporary. If he stays on this pleasure satisfaction, then he will have mental problems. In order to enter the symbolic order, the subject must overcome the desire for the original pleasure. However, although the subject can be freed from the original pleasure with the help of language, this cannot completely eliminate the original pleasure, it will also appear temporarily in other forms. This is the remainder of the original pleasure, which Lacan calls object a. The correlation between the residual pleasure of object a and different subjects is shown in Figure 3.

The existence of object a cannot solve the fundamental problem. The residual pleasure is always an empty shell. Its function is actually to cover up the alienation that people have experienced. Object a itself is a contradiction. We always want things to move according to our own consciousness, and we always hope that things are within our expectations. Although things go against our expectations in most cases, this is our pursuit of the original pleasure of the original subject and object.

The article "The Subject Construction and Role Mental Model Construction of Erotic Movies Based on Lacan's Desire Theory" was retracted in 2024. Reasons: signs of a paper mill; suspected computer-generated content; unreliable results or conclusions; concerns about the data.

On this basis, Lacan's disciple Zizek revealed the core of ideology: “The function of ideology is not to provide us with an outlet to escape reality, but to provide us with social reality itself, such a social reality. It can allow us to escape from some traumatic, real core.” That is to say, ideology itself has become the false closing button set in the elevator, which satisfies the subject's needs while covering up the real trauma. This kind of detachment between the subject and the other is the result of the ideological phantasm that guides the subject as the remainder of the original pleasure. To get rid of the false residual pleasure and move towards the true self requires the concealment and revealing of the subject spirit.

### 3.3. The Trap of Desire: Man's Desire Is the Desire of the Other

The guidance of the subject's desire by object a immerses the subject in the labyrinth of residual pleasure, and desire itself is bound to be connected with the external symbolic order. Revealing the essence of desire also brings up the question of the object of desire. Lacan's desire object is very different from Freud's desire object. Freud's desire object is a narcissistic return to the self, while Lacan's desire object is more aimed at the other. In his view, the object of human desire is the compromise and misrecognition of the capitalized Other. In Lacan's eyes, human narcissism is already a heterosexuality that misidentifies the other. The object of desire is no longer the direct object I want, and it is no longer related to me but is misidentified through the intermediary of the other. The correlation between human desire and the desire of the big other is shown in Figure 4.

Human desire is desire for the other, and Lacan regards this desire as a misrecognition of the other. We think that what we want is our desire, but the root of our desire is the other's recognition of my value. In front of desire, the other is the other, and I am still the other. The object of desire is always on the chain of signifiers, and its direction can never be fixed.

### 3.4. The Destination of Desire: The Desire of the Subject for Nothing

When the subject takes the desire of the other as the object of desire, the subject has actually completed the fantasy of the other, and this fantasy is the essence of desire. Zizek pointed out: “The desire realized in fantasy is not the subject's own desire, but the desire of the other. The formation of fantasy and fantasy is a response to the mystery of the other's desire, which determines the subject's originality. The initial question of desire is not directly ‘What do I want?' but ‘What do others ask of me? What do others see from me? How do I deal with others?'.” All are answered in the fantasy of the subject, and desire is to pursue this fantasy of answering the desires of others. The desire duration of the subject's desire for nothing is shown in Figure 5.

The article "The Subject Construction and Role Mental Model Construction of Erotic Movies Based on Lacan's Desire Theory" was retracted in 2024. Reasons: signs of a paper mill; suspected computer-generated content; unreliable results or conclusions; concerns about the data.

The order established in fantasy is inherently false, and our desire is an assumption based on it, so our desire is also false in nature. As Lacan said: “Nothing is in and out of the waltz that drives human meaning, desire is more empty than nothing, it is the remnant of the journey, like the sword of the signifier on the shoulders of the speaking subject. It is more the pure act of the signifier than the pure passion of the signified, which ceases when the living body becomes a sign, making it meaningless.” In the chain of signifiers, there is still the existence of its own meaning, and the desire, which is restrained by fantasy, itself has become a synonym for the meaningless movement of the signifier. Desire itself has no end, desire is desire for nothing, and only when the subject's life ends and becomes a symbolic symbol, the chain of signifiers of desire finally ends and becomes permanent meaninglessness.

Anyone who has experienced all these illusions and seen through the illusions of this world is desiring to become nothing and is not the subject's desire for nothingness an inner manifestation of his own subject spirit? What they want to achieve is to transcend the shackles of all symbolic orders in the world through the spirit of the subject, so that their body and mind can be truly free and transcended.

### 3.5. Subject Experience Assessment Based on Role Mental Model

Using the Likert scale, each element is divided into 5 grades on a scale of 1-5. In the evaluation process of existing erotic movies, users are guided to evaluate and score existing erotic movies, and the statistical results of user interview scores are shown in Table 1.

## 4. Discussion

### 4.1. Interpretation of Desire

Psychoanalysis has taken “desire” as one of the basic concepts since Freud [21]. Desire in Freud's theory is entangled with instinct. He regards instinct as a kind of force, which is the force and inner drive that can arouse people's behavior and divides it into two categories: life instinct and death instinct [22]. Freud believed that desire is also a kind of energy, which is in the unconscious like instinct, and desire can also cause people to act to satisfy themselves [23]. There is no strict distinction between the concepts of desire and instinct in Freud. But strictly speaking, instinct exists before desire, and desire arises from instinctual impulse.

The article "The Subject Construction and Role Mental Model Construction of Erotic Movies Based on Lacan's Desire Theory" was retracted in 2024. Reasons: signs of a paper mill; suspected computer-generated content; unreliable results or conclusions; concerns about the data.

Lacan's interpretation of desire has a new development on the basis of Freud. He uses three levels: needs, desires, and demands. This replaces Freud's instinct theory, whereby desire takes on a clearer character [24]. Lacan believes that “Needs refer to the needs of the human body and belong to the realm of physiology. Requests are requests for love, which involve a kind of human interaction. Desires are only when the object of the need is not satisfied. will arise.” From this, Lacan gave a precise definition of “desire”: “Desire is neither the satisfaction of appetite nor the demand for love, but the difference obtained by subtracting the former from the latter.” Desires arise when needs cannot be satisfied, but desires cannot be directly expressed, so desires can only be conveyed in the form of demands and through language [25, 26]. Lacan's interpretation of desire does not focus on the analysis of the content of desire; he pays more attention to the relationship between the subject's desire and being the other (social culture) [27].

When the “need” cannot be satisfied, an internal force will be formed, and the film digests and digests this force through the use of film language and certain plot settings or transformations. This force is desire. The film language mentioned here refers to the actor's body in a narrow sense, because the actor's body is the most basic visual symbol of the film language, and it is the performance and display of the body that can converge into a complete film meaning.

In a broad sense, it also includes the language and social and cultural conventions of human society. For example, the dialogue (the sound of the body on the screen) can be understood by the audience due to its universal language and plays a very important role in driving the narrative of the film.

Some common cognitions in social culture also belong to a broad language. For example, when there is a tired man walking alone in the Gobi Desert on the screen, all the audience will understand that this man is suffering from disaster and will be worried about his situation.

### 4.2. Discussion on the Expression Structure of Desire

To a certain extent, the film leaks the unconscious desire of the filmmaker, which can be seen from the way of expressing the body of the image [28]. For example, the girl who appears on the screen is a combination of an angel's face and a devil's body. Then, the filmmaker expresses his unconscious belief in “being both a child and an adult, that is, innocent and rich in experience” by shaping the girl's body. In civilized society, desire for children is forbidden, but desire for adults is allowed. Through movies, the desires of filmmakers are fictionally fulfilled. The filmmaker's disguised desire goes unnoticed, with the film being shown unharmed beneath the public visual realm. Filmmakers subtly disguise their desires through metaphors and metonymy and achieve film careers while obtaining alternative satisfaction [29].

The article "The Subject Construction and Role Mental Model Construction of Erotic Movies Based on Lacan's Desire Theory" was retracted in 2024. Reasons: signs of a paper mill; suspected computer-generated content; unreliable results or conclusions; concerns about the data.

Different desires are at different spiritual levels, and some desires can directly enter the level of consciousness and be perceived, so as to obtain direct satisfaction, such as the desire for food. However, some desires are repressed in the unconscious realm and cannot be perceived because they contradict the entire social civilization, such as sexual desire and violent desire.

Freud believed that if the repressed libido is not successfully sublimated, the stored energy will become a source of mental illness. So for the sake of individual balance, repressed desires are always looking for ways to be expressed and satisfied. Some proportions are sublimated, and the other part can only enter the consciousness system in disguised form.

Because of the inevitable gulf between the individual and the culture, between things and their representations, it is subordinate to complex pretense and intrigue. It can be seen that in order to satisfy the desire at the unconscious level, it must be expressed through many camouflage methods, so the exploration of the camouflage structure of desire is very important.

The film not only expresses the unconscious desire of the filmmaker but also more expresses the unconscious desire of the audience. The audience's interpretation of the movie has a desire component, and the pleasure of watching a movie actually comes from the satisfaction of the audience's unconscious desire [30]. Every audience has a subconscious desire for a sexual object, and this desire prompts him to possess it, but social civilization suppresses this desire [31]. Therefore, the audience is forced to give up the pursuit of this sexual object that cannot be obtained. The audience actually replaces the hand with the eyes and the stroking with the watching, so that their own desires can be satisfied.

### 4.3. Alienation of the Subject of Desire

The filmmaker expresses desire as both subject and object at the same time. As an object of desire, filmmakers choose ways to create films that are recognized by society and culture, such as expressing the virtues recognized by society and culture on the subject or expressing condemnation of behaviors that are not appreciated by society and culture [32]. As the subject of desire, filmmakers are dominated by their own real desires and will also express some desires that are not recognized by society and culture. Therefore, the film is always torn between two polar desires. The audience is also a contradictory synthesis of desire object and desire subject. On the one hand, audiences will not like films that fully conform to social and cultural ideals. On the other hand, audiences will not fully accept films that completely rebel against social and cultural ideals [33].

The article "The Subject Construction and Role Mental Model Construction of Erotic Movies Based on Lacan's Desire Theory" was retracted in 2024. Reasons: signs of a paper mill; suspected computer-generated content; unreliable results or conclusions; concerns about the data.

The movie throws a lot of images to the audience, and through the temptation of formal beauty, the social and cultural desires are rooted in the audience's subconscious, and we can clearly see the strong influence of social culture on human desires. These women are all beautiful and intelligent, but in fact, they are just vase-like supporting roles in the narrative structure of the film [34]. The film is more seductive in order to attract the attention of male audiences, and these female figures exist for the men on and off the screen. Therefore, what the film conveys is the desire of a patriarchal society. The audience is moved by the wonderful film and, in fact, has subtly accepted the desire conveyed by the film [35].

### 4.4. Surplus Desire and Surplus Pleasure

Lacan believes that “the absence of desire makes up for the absence of the original desire object in the form of remnants when the subject enters the symbolic period through the mirror phase.” Because of its high simulation, the film replaces the twisted board as the object of the adult's remaining desire perfectly and truly makes up for the absence of the audience's desire object [36].

The film incorporates the body: the actor's body is inside the screen; the audience's body is outside the screen but inside the film. The unique body immersion of the movie purifies the desires in the audience's body and makes up for the lack of desire in real life [37]. Therefore, the movie is the satisfaction of the audience's residual desire, and this residual desire is not the satisfaction of reality. The pleasure brought by the simulation of this desire is called residual pleasure, and the audience obtains a huge imaginative pleasure in the process of watching the movie [38].

The film is only a substitute for the object of the audience's desire, and the body in the film serves as the illusion of the audience's desire. This illusion is extremely perfect but far away from the audience. It can be said that the perfect image body is not only a kind of satisfaction for the audience's remaining desires but also a kind of harm to the audience's remaining desires [39]. Because what the movie provides to the audience is an alternative pleasure, a residual pleasure, not a real pleasure. There is a distance that can never be eliminated between the residual pleasure and the real pleasure, which also provides the filmmakers with the potential energy of creation and the passion of fantasy and also leaves a huge space for the expression of desire for the film [40].

The article "The Subject Construction and Role Mental Model Construction of Erotic Movies Based on Lacan's Desire Theory" was retracted in 2024. Reasons: signs of a paper mill; suspected computer-generated content; unreliable results or conclusions; concerns about the data.

The body in the film acts as an illusion of the audience's desire. This illusion is extremely perfect but far away from the audience. It can be said that the perfect image body is not only a kind of satisfaction for the audience's remaining desires but also a kind of harm to the audience's remaining desires. Because what the movie provides to the audience is an alternative pleasure, a residual pleasure, not a real pleasure. There is a distance that can never be eliminated between the residual pleasure and the real pleasure, which also provides the filmmakers with the potential energy of creation and the passion of fantasy and also leaves a huge space for the expression of desire for the film.

## 5. Conclusion

Lacan's desire theory makes an in-depth analysis of desire from the perspective of psychoanalysis. In his view, desire is generated in the gap between needs and requirements. It is a constant transformation of the chain of signifiers, an endless and meaningless cycle. To enter the symbolic order, one must ensure a balance between desire and the other. On the other hand, human desires are satisfied with the desires of others because of the object a that remains in the individual's infancy, and it is precisely because of object a that they are satisfied with ideological fantasies. In terms of desire itself, Lacan even put forward the famous thesis that “man's desire is the desire of the big other.” The desire devil of the big other makes the individual fall into the trap of desire. The essence of desire is that one realizes that desire is nothing but an illusion. Then, the subject will jump out of the snare of desire, and the subject himself will be liberated by breaking through the shackles of desire.

## Figures and Tables

**Figure 1:** The cognitive process of the subject of erotic movies.

**Figure 2:** The influence of the Lacanian unconscious on the subject.

**Figure 3:** The correlation between object a's residual pleasure and different subjects.

**Figure 4:** The correlation between human desire and the desire of the big other.

**Figure 5:** The duration of the desire of the subject's desire for nothing.

**Table 1:** Subject experience evaluation of existing erotic movies.

Hierarchy	Specific issues	Score
Usefulness	Suit one's needs	3.9
Reliability	Data is relatively safe	4.1
Availability	Better stability	4.7
Ease of use	Interactive operation is better	4.3
Pleasure	Satisfied overall	4.0

The article "The Subject Construction and Role Mental Model Construction of Erotic Movies Based on Lacan's Desire Theory" was retracted in 2024. Reasons: signs of a paper mill; suspected computer-generated content; unreliable results or conclusions; concerns about the data.

## Data Availability

The data used to support the findings of this study are available from the corresponding author upon request.
